RETRACTED

# The absence of MyD88 has no effect on the induction of alternatively activated macrophage during *Fasciola hepatica *infection

**DOI:** 10.1186/1471-2172-12-63

**Published:** 2011-11-11

**Authors:** HongLin Luo, Weiyi Huang, Dongying Wang, Haoju Wang, Kui Nie

**Affiliations:** 1 Laboratory of Infection & Immunology Research, College of Animal Science & Technology, Southwest University, Chongqing, China; 2 Parasitology department, College of Animal Science & Technology, Guangxi University, Nanning, China; 3 ENVA, UMR BIPAR, Ecopham, Ecole Nationale Vétérinaire d'Alfort, Maisons-Alfort, France

## Abstract

**Background:**

Alternatively activated macrophages (AAMϕ) play important roles in allergies and responses to parasitic infections. However, whether signaling through toll-like receptors (TLRs) plays any role in AAMϕ induction when young *Fasciola hepatica *penetrates the liver capsule and migrates through the liver tissue is still unclear.

**Results:**

The data show that the lack of myeloid differentiation factor 88 (MyD88) has no effect on the AAMϕ derived from the bone marrow (BMMϕ) *in vitro *and does not impair the mRNA expression of arginase-1, resistin-like molecule (RELMα), and Ym1 in BMMϕs. The Th2 cytokine production bias in splenocytes was not significantly altered in *F. hepatica*-infected mice in the absence of MyD88 *in vitro *and in the pleural cavity lavage *in vivo*. In addition, MyD88-deficiency has no effect on the arginase production of the *F. hepatica *elicited macrophages (Fe Mϕs), production of RELMα and Ym1 proteins and mRNA expression of Ym1 and RELMα of macrophages in the peritoneal cavity 6 weeks post *F. hepatica *infection.

**Conclusions:**

The absence of MyD88 has no effect on presence of AAMϕ 6 weeks post *F. hepatica *infection.

## Background

Macrophages are highly plastic cells that respond to diverse environments by altering their phenotype and physiology [1,2] and play important roles in both innate and adaptive immunity. Currently, macrophages are classified under two phenotypes, classically activated macrophages (CAMΦ) and alternatively activated macrophages (AAMΦ). CAMΦ are induced by interferon-gamma (IFN-γ) and lipopolysaccharide (LPS), whereas induction of the AAMΦ phenotype is associated with various stimuli, such as IL-4/IL-13, IL-10, immunocomplexes, and glucocorticoids [2]. The most widely studied stimuli for generating AAMΦ is treatment with IL-4/IL-13 [1,3]. Although IL-4/IL-13 signaling are essential to the presence of AAMΦ and both cytokines have many overlapping activities on macrophages, they exhibit distinct functions because of their specific receptor subunits aside from their shared common alpha chain [4]. However, this does not alter the fact that a Th2-dominated environment is critical for AAMΦ induction [5-7]. All helminths have been demonstrated to induce profound Th2 responses, which are characterized by the production of IL-4, IL-5, IL-9, IL-10, and IL-13 by CD4^+ ^T cells [8], and this Th2-dominated cytokine profile is associated with the presence of the AAMΦ phenotype (such as in *Schistosoma mansoni *[9], *Taenia crassiceps *[10], *Brugia malayi *[11], *Heligmosomoides polygyrus *[12], *Nippostrongylus brasiliensis *[13], and *F. hepatica *infection [14,15], and so forth). AAMΦ are increasingly recognized as a key effector arm of the Th2 immunity, but their real function in various helminth infections has not been illustrated and is likely to be diverse. However, discovery of molecular markers of AAMΦ, such as mannose receptor (CD206), IL-10, arginase -1 (instead of inducible nitric oxide), resistin-like molecule (RELMα), and Ym1 [6,16-19], made the identification of AAMΦ possible. Among them, three most abundant IL-4/IL-13 dependent genes: Ym1, a member of the family 18 chitinases family but with no chitinolytic activity [20], RELMα, was described as FIZZ1 [21], and is identified as a cysteine-rich molecule associated with resistin that is involved in glucose metabolism [22]. Arginase 1 plays a role in the regulation of nitric oxide (NO) production by competing with iNOS for substrate L-arginine [23], suppression of T cell responses via L-arginine depletion [24] and has been currently accepted as a molecular signature for AAMΦ. However, the functions of AAMΦ in helminth infections have not been fully illustrated. Questions such as whether AAMΦ promotes helminth killing or expulsion, whether alternative activation requires anti-worm effector function, or whether signaling TLRs play a role in AAMΦ induction, have not been fully answered.

RETRACTED

In the current study, the role of TLRs in AAMΦ induction during *F. hepatica *infection, which has been observed to produce Th2-dominated responses in both mice and the natural ruminant hosts [14,15] is investigated using MyD88-deficient mice.

TLRs are pattern recognition receptors (PRRs) that recognize different pathogen-associated molecular patterns (PAMPs) [25]. TLR signaling is mostly MyD88-dependent [26,27] except for TLR3 signaling, which requires a TRIF adaptor [26,27]. Mice lacking MyD88 cannot respond to LPS [28]. The absence of MyD88 has been demonstrated to have no effect on the augmentation of Th2 responses [29,30], which indicates that Th2 responses are elicited in a MyD88-independent manner. However, contrary results have also demonstrated that TLR signaling plays a role in Th2 responses [31]. Aside from the required Th2 environment, especially with IL-4/IL-13, the determinants of the AAMΦ phenotype remain unclear. For *F. hepatica *infection, whether TLR signaling is required for AAMΦ induction is unknown. Therefore, whether AAMΦ could be induced without MyD88 and whether TLR signals affect AAMϕ activation were investigated.

## Results

### Lacking of MyD88 has no impact on the presence of AAMΦ derived from bone marrow

To determine whether MyD88 signaling is required for AAMΦ induction, investigations were made to determine whether BMMϕ, cultured from both WT and MyD88 knockout mice, could be activated through this approach. This is based on the fact that arginase-1 upregulation, which is generally associated with Th2 cytokines, such as IL-4 [32], is a feature of AAMΦs. As a control, iNOS, the enzyme associated with CAMΦs, was also detected [33]. BMMϕs were treated with LPS and IFN-γ, either together or separately, or with media alone for 20-24 h after overnight treatment with or without IL-4. Subsequently, arginase-1 and iNOS enzyme activity were measured (Figure 1). The results show both WT and MyD88-/- BMMϕ cells displayed arginase activity in response to IL-4 compared with the cells without IL-4 stimulation even though no statistically significant differences were found between groups (Figure 1A). WT BMMϕs treated with LPS also exhibited arginase activity and were absent in MyD88-/- mice. iNOS activity was monitored by measuring nitrite concentrations in the BMMϕ supernatant fluids using the Greiss reagent. The results show that WT BMMϕs (with or without IL-4 stimulation) produced nitrite when stimulated with LPS alone and with IFN-γ. A synergistic effect was observed on the iNOS activity with further upregulation when treated with both LPS and IFN-γ compared with LPS or IFN-γ treatment alone (Figure 1B). MyD88-/- BMMϕ showed similar trend with WT BMMϕ on NO production. However, almost no NO was detected upon stimulation with LPS alone compared with WT BMMϕs. Moreover, NO could be produced via pretreatment with IL-4 followed by stimulation with LPS alone. Treatment with IFN-γ alone had no effect on NO production (in both WT and MyD88-/- BMMϕ) even with IL-4 treatment (Figure 1B).

**Figure 1:** **The absence of MyD88 has no effect on the AAMϕs derived from bone marrow *in vitro***. The BMMϕ were treated with or without IL-4 followed by the stimulation with LPS and IFN-γ together or separately for 12-24 h. (A). The urea concentration represents the arginase activity after the stimulation. (B). The nitrite concentration is shown as a measure of iNOS activity produced by the BMMϕs. Five mice were tested per group. Results are compiled from three independent experiments.

RETRACTED

### MyD88-deficiency of has no effect on arginase-1, RELMα, and Ym1 expression in BMMϕs

To ascertain further the phenotype of the AAMϕs elicited by the *F. hepatica *infection, the gene expression of AAMϕ markers arginase-1, RELMα, and Ym1 in BMMϕ were measured via real-time reverse transcriptase polymerase chain reaction (RT-PCR). The results show no deficiency in AAMϕgeneration in the MyD88-/- animals. Figure 2 shows that arginase-1 expression in MyD88-/- BMMϕ treated with IL-4 was lower than that of WT BMMϕ, and no expression on both untreated WT and MyD88-/- BMMϕ. The expression profiles of both RELMα and Ym1 in the BMMϕs show similar trends with higher levels on the MyD88-/- BMMϕ treated with IL-4; however, no statistically significant differences were found (Figure 2).

**Figure 2:** **MyD88-deficiency did not impair arginase-1, RELMα, and Ym1 expression in BMMϕs**. mRNA was extracted and real-time RT-PCR for arginase-1, RELMα, and Ym1 expression was carried out to examine AAMϕ generation. The black bars represent the mRNA expression in mice treated with IL-4. The mRNA expression is shown as a percent of the positive control sample and β-actin was used to normalize the experiments. Results are compiled from three independent experiments.

### The Th2 cytokine bias is not significantly altered in *F. hepatica*-infected mice in the absence of MyD88 *in vitro *and *in vivo*

Ascertaining any effects on the overall Th2 response in *F. hepatica*-infected mice is essential before determining the effect of MyD88 knockdown on macrophage activation *in vivo*. Consequently, the Th2 cytokines IL-4, IL-5, IL-10, and IL-13, together with IFN-γ, a marker of Th1 response, were monitored in the supernatant fluids of cultured splenocytes treated with media, anti-CD3, or FhAg (Figures 3A-3E). The results showed that all Th2 cytokines were elevated on FhAg stimulation in the infected WT mice and were further increased in the MyD88-/- infected mice, although no statistically significant difference was found between the WT and MyD88-/- infected mice. In contrast, the Th1 response, as measured with IFN-γ decreased significantly upon stimulation with FhAg or anti-CD3 but not media in the infected MyD88-/- mice compared with the WT infected mice (Figure 3E). Meanwhile, the thioglycolate-injected WT and MyD88-/- mice exhibited low levels of both Th1 and Th2 compared with their infected counterparts. The local cytokine production in the PEC supernatant fluid (Figures 4A-4E) was also measured. Significantly higher IL-4 levels were observed in the MyD88-/- infected mice compared with both the WT and the WT-infected mice (Figure. 4 A). Similar trends were seen in cytokine IL-5 and IL-13 (Figures 4B and 4C). However, no statistically significant difference in IL-10 production was found between the WT and MyD88-/- mice in both the thio and infection treatments. In contrast, the IFN-γ in the both MyD88-/- thio and the MyD88-/- infected mice significantly decreased compared with that in THE *F. hepatica-*infected WT mice. Overall, these results show that the Th2 response is not impaired in *F. hepatica-*infected MyD88-/- mice both *in vitro *and *vivo*.

RETRACTED

**Figure 3:** **The Th2 cytokine production bias in splenocytes was not significantly altered in the *F. hepatica*-infected mice in the absence of MyD88 *in vitro***. Splenocytes collected from C57BL/6 mice were stimulated with media alone, anti-CD3, or *F. hepatica *antigen (FhAg) for 72 h. The levels of IFN-γ, IL-4, IL-5, IL-10, and IL-13 in the supernate were measured indirectly via ELISA. The statistical significant differences were determined via one-way ANOVA followed by a Kruskal-Wallis test. *p < 0.05. Five mice were tested per group. Results are compiled from three independent experiments.

**Figure 4:** **The Th2 cytokine production bias in the pleural cavity lavage was not significantly altered in the MyD88-deficient *F. hepatica*-infected mice**. Peritoneal exudate cells (PEC) were collected from the C57BL/6 mice and were treated with media alone, anti-CD3, or *F. hepatica *antigen (FhAg) for 72 h. The levels of IFN-γ, IL-4, IL-5, IL-10, and IL-13 in the supernate were measured indirectly via ELISA. Statistical significances were determined via one-way ANOVA followed by a Kruskal-Wallis test. * *p *< 0.05 and ** *p *< 0.01. Five mice were tested per group. Results are compiled from three independent experiments.

### MyD88-deficiency did not affect the arginase production of the *F. hepatica*-elicited macrophages in PECs

To determine whether MyD88-deficiency affects production in macrophages recruited in PEC, the arginase activity levels were measured using the purified macrophages from the PEC (Figure 5). As shown, macrophages from *F. hepatica*-infected mice produced more arginase than macrophages from the mice treated with thioglycolate, and the MyD88-/- and WT infected mice produced significantly higher arginase than the MyD88-/- thio mice, although no difference was seen between the WT thio and the WT infected mice. In addition, no significant difference in arginase levels was observed between the WT and MyD88-/- infected mice.

**Figure 5:** **MyD88-deficiency has no effect on arginase production of the *F. hepatica*-elicited macrophage (FeMϕ)**. Six weeks after *F. hepatica *infection, macrophages were purified from the PEC by adherence and the levels of arginase activity were measured. Thioglycolate (thio) was also injected as the control. Significant differences were determined via one-way ANOVA followed by a Kruskal-Wallis test. *p < 0.05 and ** *p *< 0.01. Results are compiled from three independent experiments.

RETRACTED

### The absence of MyD88 had no effect on RELMα and Ym1 production by cells in the peritoneal cavity after *F. hepatica *infection

We investigated whether the absence of MyD88 impairs RELMα and Ym1 expression in peritoneal lavage fluid using western blot analysis (Figures 6A and 6B) and real-time RT-PCR (Figure 7). As shown in the figure, although both the RELMα and Ym1 protein signals were detected in the WT and the MyD88-/- infected mice, no significant difference was found between these two groups. To determine whether the mRNA expression levels correlates with protein production, total RNA was extracted from purified macrophages in the peritoneal cavity and real-time RT-PCR was performed to detect RELMα, Ym1, and arginase1 mRNA expression (Figures 7A and 7B). Although WT and MyD88-/- infected mice produced detectable RELMα and Ym1, they could not be detected in the WT and MyD88-/- thio mice. No statistically significant difference in RELMα and Ym1 mRNA expression was observed between the WT and the MyD88-/- infected mice, which is consistent with the protein profiles of RELMα and Ym1 above.

**Figure 6:** **The Absence of MyD88 had no effect on the production of RELMα and Ym1 proteins by cells in the peritoneal cavity after *F. hepatica *infection**. Six weeks after *F. hepatica *infection of C57BL/6 mice, peritoneal cavity lavages were performed and western blots for RELMα (A) and Ym1 (B) were carried out on the lavage fluid. Image software was used to measure the relative concentrations of proteins on the blots.

**Figure 7:** **The lack of MyD88 has no effect on Ym1 and RELMα mRNA expression of macrophages from the peritoneal cavity**. Six weeks after *F. hepatica *infection of C57BL/6 mice, the peritoneal cavity lavages were collected and macrophages were purified. RNA extraction and real-time RT-PCR were used for detection of RELMα (A) and Ym1 (B). mRNA expression is shown as a percent of the positive control sample and β-actin was used to normalize the experiments.

## Discussion

The data demonstrates that macrophages from a chronic infection, which consequently produce Th2 type cytokines at the stage wherein young *F. hepatica *penetrates the liver capsule and migrates through the liver tissue, do not require TLR signaling for AAMΦ induction.

Like many other helminths, to establish successful chronic infections, *F. hepatica *induces Th2 responses characterized by increased IL-4, IL-5, and IL-13, activation and expansion of eosinophils, CD4^+^cells, basophils, and mast cells [8-10,13,34-39]. Simultaneously, helminths release excretory-secretory proteins (ESP) to prevent dendritic cells and macrophages from acting on TLR2 Th1-stimulating ligands such as LPS and CpG during infections [40-42]. For example, cathepsin L1 cysteine protease released by *F. hepatica *suppresses the macrophage TLR recognition of LPS [43]. However, different infective stages may develop diverse immune responses. For instance, cytotoxic natural killer (CNK) cells dominate in the peritoneal fluid of *F. hepatica*-infected rats as early as 2 days post infection (p. i.). However, the cells decreased 4 days p.i. [44]. Therefore, the experimental set-up depends on the response outcomes needed. According to the life cycle of *F. hepatica*, the juvenile flukes penetrate the liver capsule and migrate through the liver tissue at 6 to 7 weeks before entering the bile ducts. This stage is rigorous for the host because of the violent penetration and migration of flukes. In addition, most activity detections of macrophages focus on the early stage of *F. hepatica *infection [14,45,46]; thus, little is known about the AAMΦ at 6 weeks post *F. hepatica *infection, which is the reason why the AAMΦ phenotype in MyD88 deficient mice at this stage needs to be addressed.

RETRACTED

The data demonstrates that the absence of MyD88 does not impair the Th2 response in *F. hepatica-*infected mice compared with the infected WT mice when the splenocytes *in vitro *were stimulated with FhAg. Furthermore, a non-statistically significant increase toward the Th2 response was also found in between. Moreover, the *in vivo *experiments also show that IL-4, IL-5, and IL-13 on MyD88-/- infected mice were significantly higher compared with the WT and WT-infected mice. In contrast, the IFN-γ in both the MyD88-/- thio and the MyD88-/- infected mice were significantly decreased compared with that in *F. hepatica-*infected WT mice, which indicates that a Th2- dominant response was induced *in vivo*. This is consistent with the previous studies that provide evidence of elevated Th2 responses when MyD88-deficient mice were infected with *Leishmania major *[30,47], *Chlamydia muridarum *[48], or *Schistosoma mansoni *[49,50]. Similarly, MyD88 -/- mice infected with the gastrointestinal nematode *Trichuris muris *exhibited high resistance to infection and displayed an increase in IL-4 and IL-13 in cultured mesenteric lymph node cells with stimulation of *T. muris *specific antigen *in vitro *[51] compared with their WT counterparts. However, this was argued to be associated with powerful Th1 stimuli via a MyD88-dependent pathway because of the presence of commensal bacteria, which indicates the Th2 response to nematodes might be impaired because of increased Th1 response [52]. This is supported by experiments on *S. mansoni *showing that the absence of MyD88 supports Th2 responses [50]. However, in the present study, *F. hepatica *infection was not yet reported to carry any bacteria, which may mount a Th1 response. Therefore, no significant augmentation was seen in the MyD88 deficient mice. However, the Th2 response was clearly induced in the WT mice and mice lacking MyD88 with *F. hepatica *infection. As demonstrated by previous studies, Th2 response induced by helminth infections contribute to AAMΦ production (reviewed in [53]), *F. hepatica *infection may promote AAMΦ. This is supported by the fact that AAMΦ could be produced by FhAg combined with IL-4 and stimulation with FhAg together with LPS (as a stimulus for TLR4 activity) or purified protein derivative from *Mycobacterium bovis *(PPD-B, as a stimulus for TLR2 activity) in WT mice resulted in reduced NO or IFN-γ production, respectively [54]. Also, the thioredoxin peroxidase (TPX) secreted by *F. hepatica *induced the AAMΦ on cell lines *in vitro *[14,15]. Along with the present study, an implication that MyD88 deficiency is dispensable to the AAMϕ may be reached.

RETRACTED

The present study implies that MyD88 is not required for Th2 response and AAMϕ activation. In WT BMMϕ, arginase production increased on treatment with LPS, which signals through the TLR4 pathway, which is consistent with the reports that LPS helps induce the production of both arginase isoforms (arginase-1 and arginase-2) [32,55]. Further, the arginase activity in MyD88-/- BMMϕ, treated with the media, LPS, IFN-γ, or both was almost absent, indicating that this activity is MyD88-independent. In both the WT and MyD88-/- BMMϕ, arginase mRNA increased upon treatment with IL-4, which is in agreement with the reports that arginase could be induced when stimulated with IL-4 [56] Similar trends were seen in the production of RELMα and Ym1 mRNA in WT and MyD88-/- BMMϕ in response to IL-4. These findings offering further evidence that AAMϕ is induced in MyD88 deficient mice. On the other hand, NO was produced synergistically by MyD88-/- BMMϕ when stimulated with both LPS and IFN-γ together, whereas it was produced by WT BMMϕ when treated with LPS alone. The NO produced by macrophages is essential to the suppression of host cytotoxicity and its production may be MyD88-dependent or -independent. In the present study, LPS signals through the TLR4 via the IRF-3 pathway during MyD88-deficiency, resulting in an increase in IFNβ instead of iNOS. IFNβ then induces IRF-1 production, which leads to the production of NO with the help of IFN-γ. This was supported by Koide *et al*. [57], who showed that the LPS-dependent increase in iNOS mRNA expression induced by IFN-γ is attributed to the IRF-1 upregulation induced by LPS. Moreover, iNOS cannot be induced by IFN-γ alone because of the lack of IRF-1 in the absence of MyD88. However, this speculation was not yet investigated.

RETRACTED

Considering no significant difference was found in the Th2 cytokine profiles between the WT and MyD88-deficient mice, the lack of MyD88 may have affected the production of macrophages. However, the arginase activity in the macrophages from the PEC were at approximately the same level in the WT and MyD88-/- AAMϕs (Figure 5) despite both being significantly higher than those in MyD88 -/- thio AAMϕs. RELMα and Ym1 Protein expression in the peritoneal cavity were not impaired with the MyD88-deficiency (Figure 6) and the mRNA expression of both genes (Figure 7) retained the same profiles as the protein expression, respectively. However, some effects on the response to thioglycolate treatment of the MyD88-deficient mice were observed, which indicates the partial role of TLR stimulus in thioglycolate-induced macrophage phenotype. These findings may be related to the mixture of TLR ligands in thioglycolate, which might have been ignored when the actual function of thioglycolate in macrophage activation was analyzed. All of these findings support that MyD88 is not required for macrophage activation during *F. hepatica *infection.

## Conclusion

In summary, MyD88 is not required for AAMϕ induction *in vitro *and *in vivo*. In addition, the Th2 cytokine profile remained intact in the MyD88-deficient mice infected with the *F. hepatica *6 weeks post infection.

## Methods

### Mice and infection

All animal experiments were carried out in the Animal Care and Ethics Center. Female C57BL/6 mice (6-7 weeks old) were purchased from Slaccas Experimental Animal Company. MyD88-/- mice were bred at the experimental animal center and were in the 5th and 6th generation of backcross to C57BL/6 mice. All mice were raised with free access to tap water and standard rodent diet under a pathogen-free- environment. All mice were maintained based on the Institutional and National Institutes of Health guidelines.

The wild type (WT) and Myd88-/- mice with C57BL/6 background were infected orally with 45 *Faciola hepatica *metacercariae. The metacercariae were collected from miracidia-infected *Galba truncatula *snails. All mice were euthanized 10 weeks post infection and the peritoneal exudate cells (PEC) were harvested by lavaging the peritoneal cavity with 10 mL ice-cold Dulbecco's modified Eagle's medium (DMEM) (Gibco) for mRNA extraction, western blotting, and/or cytokine analysis. The spleen was used for cell culture, which was used for the detection of cytokines *in vitro*. Then, 0.6 mL of 5% thioglycolate medium (Becton Dickinson) per mice were injected as the non-Th2 polarized inflammation control.

RETRACTED

### Activation of BMMϕ

The BMMϕs from the C57BL/6 mice were harvested from the bone marrow in the femur and tibia. Macrophage differentiation was carried out based on previous literature [58]. Briefly, erythrocytes were treated with 3 mL red blood cell lysis buffer (Sigma-Aldrich) for 5 min. The cells were cultured at 5 × 10^6 ^cells per plate in DMEM with 20% Fetal Calf Serum (FCS) (GIBCO), 20% L929 supernatant, 2 mM L-glutamine, 0.25 U/mL penicillin, and 100 μg/mL streptomycin. The medium was replaced to obtain pure macrophages at six days post culture. The collected BMMϕ were stored in fresh Petri dishes for 20-24 h with or without IL-4 (25 ng/mL; BD Pharmingen) followed by treatment with LPS (100 ng/mL; *Escherichia coli *0111:B4, Sigma-Aldrich) and IFN-γ (10 U/mL; BD Pharmingen) for 20-24 h together or separately.

### Measurement of Nitric Oxide (NO)

NO was detected via nitrite accumulation in the macrophage culture media using Greiss Reagent (Sigma-Aldrich). Briefly, 100 μL of the supernatant fluid and 100 μL of 5.8% phosphoric acid (Sigma-Aldrich), 1% sulfanilamide (Sigma-Aldrich), 0.1% N-(1-naphthyl) ethylenediamine dihydrochloride (Sigma-Aldrich) were briefly mixed. The absorbance was read at 540 nm on a microplate reader. The NO concentration was determined based on a standard sodium nitrite solution curve.

### Determination of arginase activity

Arginase activity was measured according to the previous literature [23]. Briefly, 1 × 10^5 ^macrophage cells were treated with 100 μL 0.1% Triton X-100 (Sigma-Aldrich) and 100 μL of 25 mM Tris-HCL (Sigma-Aldrich). After a 30-min shaking incubation, 20 μL of 10 mM MnCl_2 _(Sigma-Aldrich) was added. Then, the cells were heated at 56°C for 10 min to activate the enzyme and 100 μL of this lysate with 100 μL of 0.5 M L-arginine (pH 9.7, Sigma-Aldrich) was incubated at 37°C for 60 min to examine the L-arginine hydrolysis. The reaction was stopped with addition of 800 μL of H_2_SO_4 _(96%)/H_3_PO_4 _(85%)/H_2_O (1/3/7, v/v/v), and 40 μL of 9% isonitroso-propiophenone (Sigma-Aldrich). The cells were then heated at 99°C for 30 min. The plates were read at 540 nm on a microplate reader. Arginase enzyme activity was determined based on a standard urea solution curve.

### Preparation of *F. hepatica *antigens

Fresh *F. hepatica *adults from infected mice were washed with phosphate-buffered saline (PBS, pH 7.3) solution. The worms were homogenized with 10 mM Tris-HCl (pH 7.2), 150 mM EDTA at 4°C and sonicated on ice for 5 min. The homogenates were centrifuged at 12,000 × g at 4°C for 1 h. The supernatant fluids were harvested as *F. hepatica *extracted antigen (FhAg). The protein concentrations were detected using a BCA protein assay kit (Invitrogen, UK).

RETRACTED

### Cell culture and stimulation

Splenic cells and PECs were cultured *in vitro*. The spleens were crushed and the cells were centrifuged at 1100 × g for 5 min, and then resuspended at 5 × 10^6^/mL. The supernatant fluid was abandoned after the addition of 3 mL of RBC Lysis Buffer (Sigma). The cells were centrifuged at 1100 × g for 5 min followed by a final re-suspension at 10^7^/mL with the addition of 10 mL of RPMI 1640. The cells were dispensed at 5 × 10^5 ^cells per well. A final volume of 200 μL of splenic cells in triplicate were cultured with FhAg (10 μg/mL), RPMI 1640 media and anti-CD3 (1 μg/mL) at 37°C in 5% CO_2 _for 48 h, followed by the addition of 10% of total volume Alamar Blue (Invitrogen, UK) for another 24 h. The plates were read at 540 nm for cell proliferation and the supernatant fluids were harvested and kept at -20°C for further cytokine analyses after centrifugation at 1100 × g for 2 min. PEC culture and stimulation were performed similar to that for the splenocytes above.

### Cytokine determination

IL-4, IL-5, IL-10, IL-13, and IFN-γ in the spleen and PEC supernatant fluid were detected by sandwich ELISA. The plates were coated with carbonate-buffered capture antibodies at 50 μL/well (the dilution factor was 1:500 for IL-4, IFN-γ and 1: 250 for IL-5, IL-10, and IL-13) and incubated overnight at 4°C. The plates were incubated in 4% BSA PBS (200 μL/well) for 2 h at room temperature in the dark, followed by addition of 50 μL/well 2-fold diluted standard antibodies (top concentration: IL-4 at 8 ng/mL; IL-5, IL-10, and IL-13 at 10 ng/mL; IFN-γ at 50 ng/mL diluted with 1% BSA PBS) in duplicate after washing. Then, 50 μL/well of the spleen or PEC supernatant samples were then added and incubated overnight at 4°C, followed by incubation in biotinylated antibodies (final dilution: IL-4, IL-5, IFN-γ at 1 μg/mL; IL-10 and IL-13 at 2 μg/mL in 1% BSA PBS) for 1 h at room temperature and AMDEX streptavidin-peroxidase (Sigma, France) at dilution 1: 6000 in 1% BSA PBS for 30 min. Finally, 50 μL/well of TMB (KPL) was added and reaction was stopped with the addition of 50 μL of 1 mM H_2_SO_4_. The absorbance was read at 450 nm.

### Relative quantification of genes

The expression of arginase-1, RELMα, and Ym-1 genes were quantified via real-time RT-PCR. Total RNA was extracted according to the manufacturer's instructions. Approximately 1 μg of the total RNA was used to synthesize cDNA using MMLV reverse transcriptase (Stratagene). Then, the relative quantification of the genes was determined using a Light Cycler (Roche Molecular Biochemicals). A cDNA (FeMϕ)-positive control sample with five serial (1:4) dilutions was used as the standard curve in each reaction. β-Actin was used to normalize the expression of the test genes. A 10 μL reaction containing 1 μL cDNA, 4 mM MgCl_2_, 0.3 mM primers, and the Light Cycler-DNA SYBR Green I mix was carried out under the following conditions: denaturation at 95°C for 40 s, annealing at 54°C for 10 s, and elongation at 72°C for 15 s, 45-55 cycles. The annealing temperature for Ym1 was set to 62°C. The primers used for light cycler PCR analysis are listed in Table 1.

RETRACTED

**Table 1:** Primers used for real-time PCR analysis

*Gene*	*Forward*	*Reverse*	*Annealing* *Temp (°C)*
Arginase1	GGTCCAGAAGAATGGAAGAGTCAG	CAGATATGCAGGGAGTCACC	54
RELMα	GGTCCCAGTGCATATGGATGAGACCATAGA	CACCTCTTCACTCGAGGGACAGTTGGCAGC	54
Ym1	TCACAGGTCTGGCAATTCTTCTG	TTTGTCCTTAGGAGGGCTTCCTCG.	62
β-Actin	GAATCCTGTGGCATCCATGAAAC	TAAAACGCAGCTCAGTAACAGTCCG	54

### Western blot analysis

Up to 20 μL of the peritoneal cavity lavage fluid was mixed with LDS sample loading buffer (NuPAGE) and heated to resolve by SDS-PAGE using 4%-12% NuPAGE gel. The proteins were transferred from the gel onto a cellulose nitrate membrane by electrophoresis at 30 V for 1 h. Then, the membranes were incubated for 1 h in 5% skimmed milk in TBS and incubated with Anti-Ym1 (produced by immunization of the mice with recombinant protein, diluted in 5% skimmed milk in TBS blocking buffer: 1/3000) and anti-RELMα (produced by immunization of the mice with recombinant protein, 1/500) antibodies separately after 1 h block, followed by incubation with goat anti-mouse IgG alkaline phosphatase conjugate (1:5000) for 8 h. Then, it was incubated with the substrate (specify) Chemi Glow (luminol/enhancer solution: stable peroxide buffer = 1:1) until the color developed. The reaction was ceased by absorption of the rest of substrates. The results were recorded using the Gel Image System (Bio-Rad). Image software was used to measure the relative concentrations of proteins on the blots.

### Statistical analysis

One-way ANOVA was applied to evaluate the statistical differences between groups. The non-parametric Kruskal-Wallis rank sum test along with Dunn's test was applied on all analyses. Differences with *P *< 0.05 were considered significant. The values are presented as mean ± SE unless otherwise stated. All graphs were made using PRISM software (version 5.0, GraphPad Software, Berkeley, CA).

RETRACTED

## List of Abbreviations

Abbreviations: AAMΦ: alternatively activated macrophages; CAMΦ: classically activated macrophages; MyD88: myeloid differentiation factor 88; TLRs: Toll-like receptors; PRRs: pattern recognition receptors; PAMPs: pathogen-associated molecular patterns; LPS: lipopolysaccharide; IFN-γ: interferon-γ; PEC: peritoneal exudate cells; FhAg: *F. hepatica *extracted antigen; ELISA: enzyme-linked immunosorbent assay; WT: wild type; MyD88-/-: MyD88 knockout.

## Competing interests

The authors declare that they have no competing interests.

## Authors' contributions

LHL conceived, designed and coordinated the study, performed the experimental work, data collection and drafted the manuscript. WDY participated in the design of the study, analysis of assay and data collection. WHJ collected parasite materials and performed biological assay, also developed methodologies for the antibody production of RELMα and Ym1. NK developed methodologies for biochemical assay and Western blotting optimization, also provided crucial reagents and advice. All authors read and approved the manuscript.
